# Challenges experienced by midwives working in rural communities in the Upper East Region of Ghana: a qualitative study

**DOI:** 10.1186/s12884-021-03762-0

**Published:** 2021-04-09

**Authors:** Peter Adatara, Philemon Adoliwine Amooba, Agani Afaya, Solomon Mohammed Salia, Mabel Apaanye Avane, Anthony Kuug, Raymond Saa-Eru Maalman, Confidence Alorse Atakro, Irene Torshie Attachie, Constancia Atachie

**Affiliations:** 1 Department of Nursing, School of Nursing and Midwifery, University of Health and Allied Sciences, Volta Region Ho, Ghana; 2 Department of Nursing, College of Health Sciences, Kwame Nkrumah University of Science and Technology, Kumasi, Ghana; 3 College of Nursing, Yonsei University, 50-1, Yonsei-ro, Seodaemun-gu, 03722 Seoul, South Korea; 4 Department of Basic Medical Sciences, School of Medicine, University of Health and Allied Sciences, Volta Region Ho, Ghana; 5 Department of Nursing, Christian Service University College, Kumasi, Ghana; 6 Department of Midwifery, School of Nursing and Midwifery, University of Health and Allied Sciences, Volta Region Ho, Ghana

**Keywords:** Midwives, Midwifery care, Experiences, Challenges, Ghana

## Abstract

**Background:**

In 2017, a total of 295,000 women lost their lives due to pregnancy and childbirth across the globe, with sub-Saharan Africa and South Asia accounting for approximately 86 % of all maternal deaths. The maternal mortality ratio in Ghana is exceptionally high, with approximately 308 deaths/100,000 live births in 2017. Most of these maternal deaths occur in rural areas than in urban areas. Thus, we aimed to explore and gain insights into midwives’ experiences of working and providing women-centred care in rural northern Ghana.

**Methods:**

A qualitative descriptive exploratory design was used to explore the challenges midwives face in delivering women-centred midwifery care in low-resource, rural areas. A total of 30 midwives practicing in the Upper East Region of Ghana were purposefully selected. Data were collected using individual semistructured interviews and analysed through qualitative content analysis.

**Results:**

Five main themes emerged from the data analysis. These themes included were: inadequate infrastructure (lack of bed and physical space), shortage of midwifery staff, logistical challenges, lack of motivation, and limited in-service training opportunities.

**Conclusions:**

Midwives experience myriad challenges in providing sufficient women-centred care in rural Ghana. To overcome these challenges, measures such as providing adequate beds and physical space, making more equipment available, and increasing midwifery staff strength to reduce individual workload, coupled with motivation from facility managers, are needed.

## Background

Maternal mortality is high. Globally, a total of 295,000 women lost their lives due to pregnancy and childbirth in 2017, with sub-Saharan Africa (SSA) and South Asia accounting for approximately 86 % of all maternal deaths. That year, the global maternal mortality ratio (MMR) was 211 per 100,000 estimated live births. However, since 2000, there has been a 38 % reduction in the MMR, reflecting about a 2.9 % decline in global MMR annually between 2000 and 2017 [1]. If the pace of progress accelerates enough to achieve the United Nation’s 2030 Sustainable Development Goals (SDGs), which include reducing MMR to less than 70 per 100,000 live births, it would save at least 1 million women worldwide [1, 2]. The MMR in Ghana is exceptionally high, with approximately 308 deaths/100,000 live births in 2017 [2]. Most of these maternal deaths occur in rural areas than in urban areas due to a higher prevalence of skilled birth attendants (74 %) in urban areas than in rural areas (43 %) [3].

Global research has concluded that midwives play a pivotal role in providing maternity care in low- and middle-income countries [4]. Previous studies show that appropriate, accessible, and equitable birth care provided by skilled birth attendants such as midwives is a strategy that is crucial in saving the lives of pregnant women and preventing morbidity [4–6]. According to the International Confederation of Midwives (ICM), “*the midwife is recognised as a responsible and accountable professional who works in partnership with women to give the necessary support, care, and advice during pregnancy, labour, and the postpartum period, to conduct births on the midwife’s own responsibility and to provide care for the newborn and the infant*” [7].

Empirical evidence shows that when midwifery care is provided by educated, trained, regulated, licenced midwives, it is associated with improved quality of care and rapid and sustained reductions in maternal and newborn mortality [6, 8]. Evidence indicates that the deaths of women during pregnancy are generally lower in countries where most women give birth utilising the services of skilled providers, including those with midwifery skills [5]. In most sub-Saharan African countries, including Ghana, birth care in rural areas is provided by trained midwives [9]. Although midwives play important roles in providing maternal health care in the rural areas of Ghana, reports from the Ghana Health Service show that out of a total of 7,677 midwives in the country, only 462 are practising in the Upper East region of Ghana [10]. Although the number of trained midwives in Ghana has improved over the years, there is an inequitable distribution of midwives across the country, with rural and low-resource areas such as northern Ghana being disadvantaged by the inequitable distribution of health workers. Empirical studies indicate that to improve access to skilled midwifery care services and reduce the burden of maternal morbidity and mortality in rural areas, there is a need to expand pre-and in-service training opportunities and increase resources to enhance the scope and quality of services that midwives can provide in rural and low-resource areas [5, 11].

Midwives are the mainstay of providing maternity care to women in the rural areas of Ghana. They provide life-saving referrals of high-risk pregnant women to hospitals and professional care for women who do not have easy access to hospitals. Studies have revealed a number of challenges to midwifery in low- and middle-income countries including low professional autonomy, unmanageable workloads, lack of resources, lack of motivation, and inadequate staffing [4, 12–14]. These studies revealed that the challenges experienced by midwives affected the quality of care they provided [4, 12–14]. Most previous studies have focused on the experiences of mothers utilising skilled birth care [15–18]. Despite the important role midwives play in maternal healthcare in rural settings, studies exploring the challenges midwives face are scarce. This study aims to provide an opportunity for midwives to share their challenges and experiences in the Bongo District of Ghana and to advise policymakers and other stakeholders. Giving these midwives a voice may lead to increased motivation and better working conditions, which in turn could better women-centred care.

## Methods

### Research design

An explorative, descriptive qualitative study design was used to explore and describe the experiences of midwives providing women-centred midwifery care in rural areas of Ghana.

### Study setting

The research was carried out in the Bongo District in the Upper East Region of Ghana. Bongo District is one of the nine districts in the Upper East Region of Ghana. The district was selected as the study setting because it is one of the most rural and deprived districts in Ghana. The district has one hospital with six health centres located throughout the district. The hospital employs one general practitioner (medical officer) and midwives to provide skilled birth care. The rest of the maternity units in the district are manned by midwives providing primary maternity care for women during pregnancy and childbirth.

### Study population and sampling strategy

In this study, 30 registered midwives were purposefully selected and asked about challenges they faced in providing care in their respective health facilities. The researchers strived to recruit a maximum variation sample to include diverse experiences in the study.

### Inclusion and exclusion criteria

The study included midwives who had three or more years of work experience in the district and were fully employed as registered midwives. We chose registered midwives because they were fully in charge of the day-to-day activities of the maternity units. Midwives who were on postretirement contracts and auxiliary midwives were excluded from the study. Additionally, midwives on rotation were excluded.

### Data collection method

Data were collected through semistructured interviews using a flexible interview guide to explore midwives’ experiences and challenges in the rural areas of northern Ghana. The interview guide was designed to suit the context of the study setting and to encourage midwives to discuss their experiences. The interviews took place in safe, quiet, comfortable, private, and mutually agreed-upon locations. Thus, participants had the opportunity to express their challenges with minimal interruption. The interviews lasted from 45 to 60 min and were recorded and then transcribed verbatim. Data collection continued until no new information was forthcoming, even with probing.

### Data analysis

A qualitative content analysis was employed to analyse data as described by Padgett [19]. There were no pre-empted themes to guide this study, so the appropriate form of analysis was inductive content analysis. The researchers read and reread the transcripts several times to make meaning of midwives’ input. Transcripts were coded after reading sentences word by word carefully to identify words or phrases that spelled out the meaning of the sentences. Before and during the coding process, the first and third authors coded the same interviews to identify and discuss differences and check for intercoder reliability. Similar words and phrases were categorised to form themes and to ensure that they were representative of the midwives’ views. The researchers discussed and agreed on the themes.

### Ethical consideration

 The Ethical Committees of the Faculty of Post Graduate Studies Committee at Nelson Mandela University approved this study (reference number: H14-HEA-NUR-30). Written informed consent was obtained from all participants after providing them with the purpose, general content, and the nature of the investigation. Confidentiality and privacy of participants’ information were ensured. Participants were also informed of their right to withdraw from the study at any particular point in time.

### Rigour

Rigour was demonstrated by the researchers’ efforts to confirm information that was discovered and to ensure that the information accurately represented the study participants’ views. Researchers followed up with respondents to verify themes suggested by the midwives’ responses and to confirm that the participant agreed with the interpretation of her responses. The researchers also purposively selected and interviewed midwives who had experienced challenges in their work. The first author met the participants before their interviews to establish rapport. Facilitative communication skills such as probing, minimal verbal responses, and clarification were used to validate the meaning of communicated messages and observations. Transcripts were read several times to develop a coding framework, which was finalised through consensus among investigators. The researchers also provided a detailed description of the study setting and methodology (COREQ criteria were used) [20].

## Results

Midwives’ years of practice ranged from a minimum of three to 10 years. Most participants provided frontline care. Emergent and often interlinking themes were identified from the narratives obtained from midwives. Five themes emerged from the individual interview transcripts regarding the challenges experienced by midwives in care delivery to rural women:

1. Inadequate infrastructure (lack of beds and physical space).
2. Shortage of midwifery staff.
3. Logistical challenges.
4. Lack of motivation.
5. Limited in-service training.

### Inadequate infrastructure (lack of beds and physical space)

One of the key themes that emerged from data analysis was inadequate infrastructure (lack of beds and physical space) to render quality care. All participants acknowledged that inadequate infrastructure, such as rooms to accommodate many labouring women, was challenging and frustrating. They further bemoaned that the chronic lack of beds affects the quality of midwifery care because women must be laid on mattresses on the floor. This means they have to always bend or squat to deliver care to these women, and that has negative health implications for the patients as well as the midwives, who have to bend and twist in painful ways. They further expressed that cases that they could handle in the facility were referred to district hospitals due to a lack of beds in the clinics. This was inconvenient to the pregnant women and their families.

“*In rural areas, we have big problems with wards and beds. Sometimes, due to inadequate rooms and beds, anytime we have more than three women in labour, we are compelled to put them on mattresses on the floor because the room can only contain three women at a time”.*

### Shortage of midwifery staff

The shortage of midwives in the district was a major issue across the facilities, as midwives lamented about this chronic shortage, which affects their ability to function effectively due to work overload. Most midwives were compelled to work for 24 -hour shifts because there was no one to take over for them so they could get some rest. They explained that working for a whole week without rest was stressful and further affected their ability to deliver care effectively.

*"In this clinic, we are only three midwives manning the maternal and child health services. We currently handle the responsibilities of about five or more midwives which is making us get stressed up…".*

Most participants also indicated that apart from working around the clock, due to the shortages of midwives in rural areas, many of them hardly take their annual leave as required by all public service workers. Some participants felt exhausted due to continued care delivery without breaks, which was causing burnout.

*“We hardly take our annual leave because of the inadequate number of midwifery staff in our facilities. I have not taken my annual leave for three years I have been posted here as a midwife”.*

### Lack of motivation

All participants in this study acknowledged that despite the workload on midwives in rural northern Ghana, they were not compensated or incentivised. The midwives felt unnoticed and that their efforts to deliver quality maternal and child health services went unrecognised.

*“I must say that it appears no one recognises our work in this remote area where there is a lot of work. I have never been paid any allowance since I started working in this remote area for almost five years now”.*

Participants indicated that although other health providers, such as doctors, are given rural allowances as incentives to accept posting to rural and deprived areas of northern Ghana, midwives are not.

*“I feel we (midwives) are unfairly treated by the Ghana Health Service or government because we are working in the most deprived and rural areas of northern Ghana. Doctors do not work in these areas, and yet we are not given any rural incentive allowances. However, medical doctors who are not working in these areas are given rural incentive allowance”.*

Almost all participants indicated that if the government wants midwives to accept postings to rural and deprived areas in northern Ghana, there is a need to implement rural incentive allowances. Midwives need to be encouraged to accept these positions in areas where they could have a significant impact in reducing maternal mortalities.

*“…If the government wants midwives to accept posting to these remote areas, then the government should introduce rural incentive allowances for midwives to encourage them to accept posting to rural areas like here (the study setting) as the government has done for medical doctors”.*

Although most participants felt unmotivated by the government and medical facility management, a few admitted that promotions and study leave with pay were granted much faster for midwives working in rural areas than those working in developed towns and cities. Some midwives still expressed great concern that although the study processes were much faster, they were not able to continue their educations due to staff shortages.

*“…However, I must say that our only advantage and motivation for working in these rural areas is that our promotions are faster than our colleagues in the towns and cities”.*

*“One good thing about working in these rural areas is that we can be allowed to go to school for further studies with pay when we work for at least two to three years…”.*

### Logistical challenges

All the participants expressed frustrations due to the lack of equipment and basic consumables. They recounted many occasions when they could not perform full iterative midwifery care to expectant mothers due to a lack of supplies. The midwives further explained that they must improvise with the few resources at their disposal while knowing that these were not the best practices. They had to improvise to save the lives of the mothers and the unborn babies. The midwives felt that they were neglected by clinic managers because they made requisitions for the necessary supplies, but their voices were not heard. Below are some narrations by midwives:

*“In this clinic, the challenge we face here is not only about beds and space to put the clients but also consumables and supplies such as gloves, liquid soap, cotton, and gauze. We have always been improvising in every procedure we perform in this clinic”.*

### Limited in‐service training opportunities

All participants acknowledged that there were limited in-service training opportunities for midwives working in rural communities to improve their knowledge and skills like their counterparts who are working in towns and cities.

*“It is a disadvantage of working in rural areas in the north. As we are working here, we are only able to attend few in-service training courses, unlike our colleagues who are in the cities who have the opportunity to attend lots of workshop training all the time”.*

Participants pointed out that although they occasionally attended workshop training organised by Ghana Health Services and other institutions, due to the shortage of midwives in rural areas, many of them could not leave work to attend those workshops.

*“I must acknowledge that workshops have been organised by Ghana Health Service and other bodies, but due to our number (a few staff), we are unable to attend most of those workshops”.*

Participants reported that apart from the fact that they are unable to attend many workshops organised by the Ghana Health Service and other organisations to improve their knowledge and skills, they also do not have the opportunity for effective mentorship and coaching by senior and experienced midwives in rural areas.

*“…Hmmm, our problems are just too many. When you are posted here, you are just on your own. There are no senior or more experienced midwives here to mentor or coach us…”.*

## Discussion

Midwives are important maternal healthcare providers in rural Ghana. This study explored and described the challenges experienced by midwives who provide maternal healthcare to childbearing women and their newborns. One of the major challenges experienced by midwives working in rural northern Ghana was inadequate infrastructure (lack of physical space and beds). Inadequate infrastructure such as wards and beds to accommodate multiple labouring women at the same time was reported as a major challenge. This greatly hindered the quality of care they were able to provide. This finding is consistent with previous studies that identified inadequate wards and hospital beds as major challenges affecting the quality of care in rural communities [11, 21]. The current study also supports findings from another recent study conducted in rural northern Ghana, where there was no physical space to admit women needing childbirth services [22]. In resource-constrained settings, women in labour will have to queue in health facilities for childbirth services due to overcrowding and share beds with other women during and after childbirth [23]. In some cases, where there were limited beds in the facilities, women would have to lie on floors or mattresses after childbirth [23, 24]. Although the health sector has seen improved infrastructure over the years, rural and low-resource areas of the country still lack adequate infrastructure to accommodate the increasing number of patients and clients seeking healthcare in the clinics.

The shortage of midwifery staff in the rural areas of Ghana remains an important issue of interest to policymakers and the government. This study found understaffing to be a serious challenge affecting quality midwifery care. To help bridge this gap, most midwives have to work overtime, while some do not even take their annual leave. According to study participants, adequate staffing is necessary for effective and adequate care in the effort to improve maternal and child healthcare. The findings of this study are consistent with the findings of previous studies conducted globally and in SSA, where insufficient personnel was the most important reason for poor conditions cited by midwives [17, 25]. For example, a study conducted in Tanzania found that the challenge midwives experienced was the shortage of midwifery personnel in the health facilities [14]. This resulted in an excessive workload that affected the quality of care provided [14]. Similarly, other studies indicate that inadequate staffing levels and increasing workloads among health professionals were a challenge across both rural and urban settings [4, 26–28]. Additionally, a study of African countries documented that inadequate staffing and excessive overtime work were found to compromise women’s safety and the midwifery staff as well [29]. Untenable workloads could place midwives in an ethical dilemma about how to prioritise care. In Malawi, nurse-midwives mentioned the daily problem of deciding who to care for, the newborn or the mother, or even another mother or another newborn [30]. The World Health Report in 2006 identified Ghana among 36 countries in SSA as one facing a health workforce crisis [31], which necessitated government intervention through the Ministry of Health (MOH) to address myriad health workforce challenges, especially among nurses and midwives. Recently, out of approximately 115,650 public sector health workers, 58 % were nurses and midwives [32, 33]. From 2008 to 2018, there was a remarkable increase in the nursing workforce of approximately 370 % [32]. Nonetheless, there exists a lingering shortage of nurses and midwives in most hospitals and clinics across the country, especially in rural settings [33, 34]. From 2016 to 2019, 40,000 trained nurses and midwives were unemployed, while health facilities across the country are in dire need of these professionals. Due to the extended credit facility agreement between the government of Ghana and the International Monetary Fund (IMF) with its associated austerity measures, most nurses who graduated from 2016 to 2018 could not be immediately employed [34].

Lack of motivation was identified as another challenge that midwives experienced in the delivery of maternity care in rural settings. The midwives felt that their efforts and sacrifices in delivering quality maternity care to improve maternal and child health were overlooked and unappreciated. They argued that some cadres of health professionals were motivated by rural incentive allowances, but they were not considered fit to also receive the allowances. Further, the midwives felt neglected because their concerns were not addressed. This finding is similar to a study by Bremnes, Wiig, Abeid, and Darj [14], where midwives felt they were not motivated to provide quality care. In the World Health Organization’s report on improving healthcare performance, supportive supervision was found to contribute to a positive performance by health workers [35, 36]. When healthcare workers are not motivated by the employer, they often lack courtesy when dealing with patients, provide poor care, and fail to treat patients in a timely manner [37]. Thus, patients’ health outcomes are critically dependent on motivation of nurses and midwives. Therefore, providing training on supportive management methods for supervisors and hospital/clinic managers is a means of increasing the level of motivation in the workplace. Health facilities that provide at least minimum allowances tend to motivate health professionals to provide quality care to patients who are more satisfied with their care [38].

The lack of basic medical equipment was another major challenge reported by midwives. The midwives were frustrated and could not deliver full iterative midwifery care due to a lack of consumables, which affected quality care. Midwives had to improvise with insufficient equipment and supplies at their disposal while knowing these were not best practices. This study finding is consistent with a study conducted in Tanzania, where midwives reported an inadequate supply of medical equipment to provide quality care [14]. A recent study in Ghana also reported inadequate medical equipment for childbirth services in rural northern Ghana [22]. The inadequacy of basic medical supplies contravenes the quality statements (statement 8) of the WHO, stipulating a positive experience for all women during pregnancy, childbirth, and postpartum care [39]. Although this lack of medical supplies affects patients receiving care, it also exposes midwives to contracting infections due to inadequate personal protective equipment. In the absence of a safe working environment, such as water for handwashing, sharps disposal, and basic medical supplies such as gloves, and limited access to post-exposure prophylaxis (PEP), midwives were exposed to HIV and other infections [40–42].

Limited in-service training opportunities were reported as a challenge experienced by midwives working in rural areas of Ghana. The global literature reported similar findings that community midwives were struggling for survival in rural areas due to a lack of limited in-service training opportunities to improve their knowledge and skills [4]. According to the WHO, a lack of adequate pre-and in-service midwifery education and professional development negatively affects preparation for the midwifery role and the building of personal autonomy, resulting in low levels of skill and confidence and poor quality of care in many countries, particularly in rural areas [9, 43]. There is a need for supportive supervision and mentoring at work, improved professional development programmes, workshops, and access to training opportunities.

## Limitations

A key limitation of this study is social desirability bias. Midwives may not report experiences that might cast them in an unfavourable light. Additionally, the sample size for this study was relatively small, and the study covered only one district in Ghana. The findings may, therefore, not be representative of the experiences and challenges of all rural midwives in the country. Nonetheless, this is an important study that explored the experiences and challenges of rural midwives, which will guide human resource management policies and decisions in the health sector of Ghana.

## Conclusions

Midwives’ experience a myriad of challenges in providing sufficient women-centred midwifery care in rural Ghana. To mitigate these challenges, measures such as providing adequate beds and physical space, making more equipment available, and increasing midwifery staff strength to reduce the workload, coupled with motivation and support from facility managers, are needed.

## Data Availability

The datasets used and/or analysed during the current study are available from the corresponding author on reasonable request.

## Abbreviations

MMR: Maternal Mortality Ratio
WHO: World Health Organisation
PEP: Post Exposure Prophylaxis
COREQ: Consolidated criteria for reporting qualitative research
IMF: International Monetary Fund
HIV: Human Immunodeficiency Virus
MOH: Ministry of Health
ICM: International Confederation of Midwives
SSA: Sub-Saharan Africa
SDGs: Sustainable Development Goals
